# Optimization and Analysis of Intelligent Accounting Information System Based on Deep Learning Model

**DOI:** 10.1155/2022/1284289

**Published:** 2022-07-31

**Authors:** Suzhen Feng, Ran Zhong

**Affiliations:** ^1^School of Accountancy, Shandong Youth University of Political Science, Jinan 250103, China; ^2^School of Economics and Management, Hebei Oriental University, Langfang 065000, China

## Abstract

Accounting information often accounts for more than 70% of an enterprise's financial report information. Accounting information is an important reference for an enterprise to make major decisions, and it is also the fundamental guarantee for an enterprise to remain invincible under the increasingly fierce business competition. With the vigorous development of enterprise informatization, traditional accounting information processing methods can no longer meet the needs of the information age. Therefore, an excellent enterprise must have a complete set of intelligent accounting information systems. How to extract the information we want from the dazzling accounting information data is a hot topic in the current financial industry. On the basis of analyzing the significance of establishing an information system, this paper creates an intelligent recognition model, which solves the shortcomings of traditional methods such as large calculation errors, time-consuming, and labor-intensive. The research results of the article show that (1) the standardized coefficients of the four influencing factors of CSR, ROE, CEO, and SCALE are relatively large, indicating that these four influencing factors have a significant impact on the development of corporate accounting and you can pay attention to these four aspects. (2) To test the performance of the article model, the experiments are compared with other models. The results show that the model proposed in this paper has the highest running success rate on the two test sets, with a success rate of more than 98%, indicating that the model in this paper has certain advantages in accounting information processing. (3) In the page response time experiment, the financial module has the shortest response time, the number of tests is 60 times, the average response time is 0.5 s, and the success rate can reach 100%. It can reach 0.8 s, and the success rate can be kept above 98%, indicating that the system can work normally. In the system operation stability test, the number of test cases designed for the financial module is 70, the number of executed test cases is 70, and the execution rate can reach 100%. This means that the system can work properly and will not fail during operation.

## 1. Introduction

In today's highly competitive business competition, enterprises must meet the complex and diverse personalized needs of the market. Enterprises must not only formulate internal management systems to ensure the normal operation of enterprises. Traditional computing methods have been gradually eliminated by society. We are in an era of informationization and intelligence. How to combine big data intelligent technology with accounting management work is a problem we need to consider. Accounting information management of an enterprise is related to the long-term development of an enterprise, so when formulating an enterprise accounting information system, we must consider many aspects. This paper proposes a rational risk assessment model that will help managers assess risk exposure due to potential threats to internal control in computer-based accounting information systems [1]. In this paper, we propose a new algorithm for risk assessment of accounting information systems using AHP [2]. The purpose of this paper is to explain how case-based reasoners can be used to support inexperienced information systems auditors in evaluating controls and making audit recommendations [3]. Based on the author's work and study experience, this paper analyzes the accounting data processing problems under the background of the times [4]. This paper analyzes the application of intelligent accounting information systems in industrial and commercial enterprises and puts forward relevant suggestions [5]. This paper studies how to identify accounting events expressed in natural language and constructs an expert system [6]. This paper studies how to identify accounting events expressed in natural language and proposes a word transfer method in accounting text analysis by introducing natural language processing technology [7]. According to the method of the Analytic Hierarchy Process, the article assigns the weights to the scheme layer and constructs a complete system of accounting information disclosure indicators in colleges and universities [8]. The article illustrates that e-accounting is a new information technology term based on the changing role of the accountant, where advances in technology have relegated the mechanical aspects of accounting to computer networks [9]. By studying the relationship between the network environment and the accounting information system and the influence of the network environment on the accounting information system, this paper proposes that the internal control measures should have a diversified development trend and proposes specific measures [10]. The article explains the development status of domestic accounting information systems and risk control methods [11]. The article summarizes the development of accounting information and accounting software in China and points out that the new changes in the future will include the birth of social responsibility accounting, the widening of accounting information, and social supervision [12]. This paper describes in detail the necessity of designing an intelligent accounting information system for enterprise accounting management [13]. This study tested the influence of intrinsic and extrinsic motivation on the behavioral intentions of Libyan SMEs to adopt accounting information systems [14]. The purpose of the article is to explain the impact of accounting environmental variables on the relationship between AIS and Iraqi performing SMEs [15].

## 2. Detailed Design of Accounting Information System

### 2.1. Introduction to Accounting Information System

The accounting information system is mainly composed of four major modules. The main module is the core part of the accounting information system. The accounting module is the basis of the information system. Interact in real-time. The budget management module realizes budget preparation through the preparation of budget drafts, enters the budget index allocation module based on the enterprise decision-making system, uses intelligent vouchers to transmit indicators to the accounting system, and uses the network to implement departmental transmission between projects. The database records all the accounting information of the enterprise and can be consulted at any time. All accounting databases are combined to form a data management system, which contains all the accounting information data of the enterprise. The functional modules of the intelligent accounting information system are shown in Figure 1.

### 2.2. The Significance of Accounting Information System

At present, big data has transitioned from the conceptual stage to the large-scale application stage. The multifunctional and globalized accounting information system based on big data is a brand-new production tool for enterprises. The application of this transformed processing mode can enable enterprises to have more powerful process optimization. Create a more dynamic organizational structure, lead new changes in the field of financial accounting, realize complex business logic management and intelligent decision-making on uncertain markets and organizational methods, and create a full ecological balance system of internal and external, horizontal and vertical dimensions, to help the leap-forward development of smart business and smart enterprises. The management concept and management work of many enterprises have undergone earth-shaking changes, and an intelligent accounting information management system has also been born in the accounting management work. Accounting management is an important part of the operation process of an enterprise. After years of precipitation, the accounting management field has developed a relatively complete and mature development model. The integration of intelligent computing technology into the work of enterprise accounting management not only greatly reduces the complexity and tediousness in the process of enterprise accounting information processing but also solves the problems of low efficiency and large errors caused by manual calculation and also liberates the labor force. In the increasingly competitive business competition, an excellent enterprise must conform to the development of society and the times, make corresponding changes, adjust the development goals of the enterprise, and formulate relevant development strategies.

## 3. System Establishment of Deep Learning Model

### 3.1. Model Establishment

To establish an enterprise indicator model, this paper adopts the following model [16]:

(1) $$\begin{array}{c} ZL_{fy}=\sum F+\sum Y+\partial_{0}+\partial_{1}*P_{fy}+\partial_{2}*M_{fy}+\cdots . \end{array}$$

Among them, *F* represents the industry in which the company is located, *Y* represents the year, and *ZL*_*fy*_ represents the change in the strategic value of the company in *F* industries and *Y* years; the changes in various accounting indicators of the company and the comprehensive benefits of the changes in the strategy of the entire company are reflected by this value, and *∂*_*i*_(*i*=1,2, ⋯, 7) represents the index coefficient corresponding to the *i*-th indicator, *P*_*fy*_ represents the investment in sales expenses, *M*_*fy*_ represents the investment in management expenses, *F*_*fy*_ represents the investment in fixed asset renewal costs, *D*_*fy*_ represents capital intensity, *l*_*fy*_ represents R&D investment, *L*_*fy*_ represents corporate financial leverage, and *C*_*fy*_ represents cloud computing ability value.

Sales expense input is as follows [17]:

(2) $$\begin{array}{c} P_{fy}=\frac{SE}{R}. \end{array}$$

Management fee input is as follows [18]:

(3) $$\begin{array}{c} M_{fy}=\frac{ME}{R}. \end{array}$$

Fixed assets renewal cost input is as follows:

(4) $$\begin{array}{c} F_{fy}=\frac{NE}{OF}. \end{array}$$

Capital intensity is as follows [19]:

(5) $$\begin{array}{c} D_{fy}=\frac{NF}{SN}. \end{array}$$

R&D investment is as follows:

(6) $$\begin{array}{c} I_{fy}=\frac{IF}{R}. \end{array}$$

Corporate financial leverage is as follows [20]:

(7) $$\begin{array}{c} L_{fy}=\frac{SD+LD+BP}{V}. \end{array}$$

### 3.2. Financial Risk Forecast

Financial risk prediction formula is [21]

(8) $$\begin{array}{c} DD\;=\frac{E\left(V\right)-D}{E\left(V\right)\sigma A}. \end{array}$$

Assuming that the price fluctuations of the real assets of the target company can obey the Wiener process, there are

(9) $$\begin{array}{c} dV_{A}=\mu V_{A}dt+\sigma_{A}V_{A}dz. \end{array}$$

The relationship between asset value and equity value can be constructed as follows [22]:

(10) $$\begin{array}{c} V_{E}=V_{A}N\left(d1\right)-e^{-rt}\times N\left(d2\right), \end{array}$$

(11) $$\begin{array}{c} \sigma_{E}=\frac{V_{A}}{V_{E}}\sigma_{A}. \end{array}$$

Expected default rate is as follows:

(12) $$\begin{array}{c} Pt=\text{prob}\left[V_{A}^{t}\leq X_{t}|V_{Z}^{0}=V_{A}\right]. \end{array}$$

Company asset value is as follows:

(13) $$\begin{array}{c} \ln\;Vt_{A}=\ln\;V_{A}+\left[\mu -\frac{\sigma_{A}^{2}}{2}\right]\tau +\sigma_{A}\sqrt{\tau \varepsilon }. \end{array}$$

Final default rate is as follows:

(14) $$\begin{array}{c} P_{t}=N\left[\frac{\ln V_{A}/X_{t}+\left(\mu -\sigma_{A}^{2}/2\right)\tau }{\sigma_{A}\sqrt{\tau }}\right]. \end{array}$$

The evaluation index of enterprise financial risk is as follows [23]:

(15) $$\begin{array}{c} X=\left(X_{1},X_{2},\cdots ,X_{p}\right). \end{array}$$

Linear combination of evaluation metrics is

(16) $$\begin{array}{c} \hat{P}=W_{0}+W_{1}X_{1}+W_{2}X_{2}+\cdots +W_{p}X_{p}, \end{array}$$

in

(17) $$\begin{array}{c} W^{*}=\left(W_{0},W_{1},W_{2},\cdots ,W_{P}\right), \end{array}$$

(18) $$\begin{array}{c} X^{*}=\left(X_{1},X_{2},\cdots ,X_{p}\right). \end{array}$$

Financial risk prediction model is as follows [24]:

(19) $$\begin{array}{c} P=\frac{\exp\left(W_{0}+W_{1}X_{1}+\cdots +W_{p}X_{p}\right)}{1+\exp\left(W_{0}+W_{1}X_{1}+\cdots +W_{p}X_{p}\right)}. \end{array}$$

## 4. Simulation Experiments

### 4.1. Model Construction

In order to find out the factors that affect the development of corporate accounting, the experiment selected 11 secondary indicators as impact factors and recorded the data of each impact factor from 2014 to 2018, so as to determine the important indicators that affect the development of corporate accounting. The value of the standardization coefficient is an important reference factor for determining the impact factor and the development degree of enterprise accounting. The larger the coefficient value, the more significant the degree of influence. The specific experimental operation is as shown in Figure 2. The definition of factor variables is described in Table 1.

According to the experimental data in Table 2, in 2014, the standardized values of 11 secondary indicators were all 1. Since 2015, the standardized values of each factor began to change. In 2015, the standardized coefficient of the ownership structure was 3.75, which is 11 items. The highest one of the test indicators indicates that the ownership structure has a greater impact on accounting information. The standardized coefficient of operational management independence is 0.1, which is the lowest of the test indicators, indicating that operational management independence has the lowest impact. From 2016 to 2018, the standard coefficients of company size and region are all higher than 1.0, indicating that the two independent variables have a relatively large degree of influence. The description of the impact factors of the secondary indicators is shown in Table 3 and Figure 3.

According to the data in Table 3, in 2014, the standardization coefficient of enterprise nature reached 0.95, indicating that the influence factor of enterprise nature was the largest. From 2015 to 2016, the standardized coefficient decreased, and the coefficient reached 1 in 2018. In 2015, except for the AREA coefficient, which reached 1 after that, the other coefficients are all less than 1, indicating that except for the region where the influence factor of the enterprise is relatively large, other influence factors have no significant influence on the development of the enterprise. In 2016, the standard coefficient of company size exceeded 1. From 2017 to 2018, the standardized coefficients of many indicators exceeded 1, indicating that these influencing factors have an increasingly significant impact on enterprise development.

### 4.2. Model Comparison Study

In order to test the performance of the accounting recognition model established in the article, the experiment will run the model and the other two models on different test sets and record the experimental results. Model evaluation classification is the last step in building a model; it can effectively help us choose an excellent classifier and improve its performance and plays a very important role. Generally speaking, the training set is used to evaluate the parameters of the model, so that the model can reflect the reality and then predict the future or other unknown information, and the test set is used to evaluate the prediction performance of the model. The experimental results under the two different test sets are as shown in Figure 4. The model evaluation indicators are shown in Table 4.

According to the data in Table 5, we can conclude that after the training set runs, the correct rate of the model proposed in this article can reach 94.8%, and the accuracy rate can reach 98.23%, which is the highest among the test models. The correct rate is 84.95%, and the accuracy rate is 94.71%, which is the lowest among the test models. The correct rate of the decision tree recognition model is 88.87%, and the sensitivity is 93.36%. The detection results are in the model proposed in the article and the support vector machine recognition model in between.

According to the above model test results in Figure 5 and Table 6, the running accuracy of the model in the training set and the test set is 94.80% and 92.23% respectively, and the running accuracy in the training set and the test set is 81.95% and 92.23% respectively. The accuracy rate is 93.21%. The correct rate of the decision tree recognition model is 88.87% in the training set and 86.14% in the test set. Although the performance of the three detection models is reduced to a certain extent after the test set is run, the detection value of the model in this paper is still the highest among all detection models. The experimental results also show that the detection efficiency of the model proposed in this article is optimal whether it is in the training set or the test set.

### 4.3. System Test

System testing is to test whether the system can work normally under a certain load [25]. The performance test of the intelligent accounting information system based on the deep learning model studied in this paper is mainly tested from the two indicators of page response time and system operation stability. The method of page response test is to record the system response time under different test times and then observe the response time and operation stability of the system by continuously increasing the number of tests and the ratio of numbers. The components of intelligent accounting information are shown in Table 7

#### 4.3.1. Page Response Time Test

According to the above experimental results in Table 8 and in Figure 6, the average response time will increase with the increase of the number of tests. The average response time of the financial part is the lowest among all the test modules. When the number of tests is 130, the average response time of the financial part is 1.2 seconds; the average response time of the purchase, sale, and storage part is 1.5 seconds, and the average response time of the management analysis part is 1.8 seconds. The management analysis part contains a huge database, so the response time is the longest, and the response time of the purchase, sale, and storage part is between the financial part and the management analysis part. Moreover, the execution success rate of the three modules has remained above 98% (Table 9).

#### 4.3.2. System Operation Stability Test

According to the execution rate test of the system in Figure 7, we can know that when the number of design test cases is 140, the number of executed use cases of the financial module is 140, the number of executed use cases of the purchase, sale, and storage module is 139, and the number of executed use cases of the management analysis part is 138. The execution rates of the three modules are kept above 98%, close to 100%, indicating that the system can operate normally.

## 5. Conclusion

Applying the processing mode transformed by intelligent computing can enable enterprises to have more powerful process optimization, create a more dynamic organizational structure, promote new changes in the field of financial accounting, and realize complex logical management of business and business operations in uncertain markets and organizational methods. Intelligent decision-making, as well as building a comprehensive ecological balance system of internal and external, horizontal, and vertical dimensions, helps smart businesses and smart enterprises to develop forward. The model proposed in this paper solves the problems of long calculation process and high error rate in the human computing process, and the model has a short response time and a high success rate, but the model still has some shortcomings. The model of this paper is to calculate only the accounting information data of a certain enterprise, and the calculation sample capacity is small. In future research work, the calculation capacity should be increased. Accounting management is a very complex task. In the process of accounting work, there will be many accounting calculation methods and related systems that cannot be explained clearly. The relevant departments of the enterprise should pay attention to revising the relevant policies of accounting management. Effective calculation of accounting information will reduce the occurrence of any illegal operations, thereby promoting the long-term development of enterprises. The construction of the new accounting information system is the result of the development of science and technology of the times. The integration of big data and accounting information processing is a new development trend. Enterprises should seize the opportunity and strive to improve their own development deficiencies. The enterprise accounting information system under big data will develop better and better and can adapt to the pace of scientific and technological development and form an accounting information system with Chinese characteristics in the process of continuous development. Enterprises need to develop and progress. The traditional audit method is inefficient and consumes a lot of manpower and material resources. Before auditing the company's financial statements, auditors can use the identification model in this study to test the possibility of accounting information distortion, clarify the key points and doubts of the audit, form a preliminary evaluation, and then determine the audit scope and audit scope. The review process is a procedure to improve the quality of accounting information audit.

## Figures and Tables

**Figure 1:** System function module.

**Figure 2:** Standardized data statistics for each factor.

**Figure 3:** Statistics of factors affecting the level of accounting information disclosure.

**Figure 4:** Statistics of model evaluation results.

**Figure 5:** Statistics of model evaluation results.

**Figure 6:** Average response time curve.

**Figure 7:** Execution test case statistics.

**Table 1:** Factor variable definition description table.

First-level indicator	Secondary indicators	Representative symbol	Definition explanation
Company financial variables	Financial leverage	LEV	Measure the financial risk of the company by the company's asset-liability ratio
	Roe	ROE	Reflect the company's profitability

Company characteristic variables	Company size	INSIZE	The logarithm of the company's total assets
	Your area	AREA	East, middle, and west are represented by 3, 2, and 1, respectively

Corporate governance variables	Board size	SCALE	Expressed by the number of board members
	Operational management independence	CEO	It is represented by the combination of the chairman and the general manager
	Shareholding structure	HERF5	Expressed in the herfind index
	Enterprise nature	NSH	1 for domestic holdings, 0 for the rest

External environment variables	Government intervention	CSR	1 for publishing social responsibility report, 0 for not publishing
	Media attention	VIZIBILITY	Select the financial media attention related to the industry to which the company belongs
	Firm influence	BIG	Indicated by firm ranking, the top ten firms take 1, otherwise take 0

**Table 2:** Standardized data of each factor.

Index	2014	2015	2016	2017	2018
EDI	1.00	0.13	0.46	0.17	1.25
LEV	1.00	0.34	0.70	0.61	1.38
ROE	1.00	0.37	0.75	0.57	0.68
INSIZE	1.00	1.05	1.20	1.10	1.29
AREA	1.00	0.50	1.41	1.50	1.33
SCALE	1.00	0.90	1.10	1.48	1.98
CEO	1.00	0.10	0.40	0.6	0.80
HERF5	1.00	3.75	3.38	0.63	0.70
NSH	1.00	0.89	0.53	0.84	1.05
CSR	1.00	0.65	0.82	0.89	0.92
VIZIBILITY	1.00	0.15	0.34	1.47	2.38
BIG	1.00	0.44	0.63	1.25	0.56

**Table 3:** Description of accounting information impact factors.

Index	2014	2015	2016	2017	2018
EDI	0.73	0.09	0.33	0.12	0.89
LEV	0.59	0.20	0.41	0.36	0.81
ROE	0.29	0.11	0.22	0.41	0.20
INSIZE	0.89	0.95	1.12	1.30	1.73
AREA	0.20	1.00	0.82	1.25	1.33
SCALE	0.89	0.86	0.92	1.34	1.65
CEO	0.05	0.10	0.02	1.00	0.40
HERF5	0.08	0.30	0.27	0.45	0.56
NSH	0.95	0.85	0.50	0.80	1.00
CSR	0.05	0.25	0.45	0.89	0.50
VIZIBILITY	0.69	0.15	0.24	1.53	2.38
BIG	0.80	0.35	0.50	1.00	0.45

**Table 4:** Evaluation index table.

	Formula	Definition
Accuracy	*PPV*=*TP*/(*TP*+*FP*)	Indicates the proportion of the model identified correctly among all results identified by the model as correct samples
Sensitivity	*TPR*=*TP*/(*TP*+*FN*)	Indicates that the model recognizes the correct proportion in the true value of the sample
Specificity	*TNR*=*TN*/(*TN*+*FP*)	Indicates that the model recognizes the correct proportions in which the true value is negative

**Table 5:** Training set model evaluation result table.

Recognition model	Correct rate (%)	Accuracy (%)	Sensitivity (%)	Specificity (%)
Deep learning recognition model	94.80	98.23	96.15	76.32
Support vector machine recognition model	84.95	94.71	87.76	64.71
Decision tree recognition model	88.87	93.75	93.36	60.53

**Table 6:** Evaluation effect of the test set model.

Recognition model	Correct rate (%)	Accuracy (%)	Sensitivity (%)	Specificity (%)
Deep learning recognition model	92.23	97.14	95.56	75.23
Support vector machine recognition model	83.21	93.89	86.22	63.79
Decision tree recognition model	86.14	92.78	92.46	60.48

**Table 7:** Components of intelligent accounting information system.

Component	Function
Financial section	Mainly responsible for the company's daily financial work and financial budget, accounting and financial management, and fundraising, etc., early warning and monitoring of financial risks, and guiding the company's business activities through financial data analysis
Purchase and sale part	According to the needs of the enterprise, in order to solve the problems of confusing accounts, inaccurate inventory, and untimely information feedback, the purchase, sale, and storage system integrates procurement, sales, inventory management, and receivable and payable management, providing order, procurement, sales, the management of returns, inventory, current invoices, current accounts, salesmen, etc., helps enterprises handle daily invoicing and inventory business, and provides rich real-time query and statistical functions
Management analysis section	Management analysis can make full use of the historical data and other relevant information provided by financial accounting, use certain mathematical methods to process them scientifically, conduct scientific forecasting and analysis for business operations, and help leaders at all levels to make decisions accordingly. Correct decision analysis

**Table 8:** Page response time test results.

Testing frequency	60	70	80	90	100	110	120	130
Financial section	0.5	0.6	0.7	0.8	0.9	1.0	1.1	1.2
Purchase and sale part	0.8	0.9	1.0	1.1	1.2	1.3	1.4	1.5
Management analysis section	1.1	1.2	1.3	1.4	1.5	1.6	1.7	1.8

**Table 9:** System operation stability test.

Design test cases	70.00	80.00	90.00	100.00	110.00	120.00	130.00	140.00
Financial section	70.00	80.00	90.00	100.00	110.00	120.00	130.00	140.00
Purchase and sale part	68.00	77.00	88.00	99.00	109.00	119.00	129.00	139.00
Management analysis section	67.00	76.00	87.00	98.00	108.00	118.00	128.00	138.00

## Data Availability

The experimental data used to support the findings of this study are available from the corresponding author upon request.
